# The Protection Mechanism of Personal Health Information in the Digital Economy Environment

**DOI:** 10.1155/2022/2314468

**Published:** 2022-06-13

**Authors:** Nan Liu, Shiyong Chen

**Affiliations:** ^1^School of Law, Southwest Medical University, Luzhou 646000, Sichuan, China; ^2^School of Marxism, Southwest Medical University, Luzhou 646000, Sichuan, China

## Abstract

With the application of big data technology in the medical field, personal health information is experiencing unprecedented challenges while showing great value. Opportunities and risks are like two sides of the same coin, and the rapid development of science and technology has not only brought valuable opportunities, but also made modern society seem to have developed into a risk society. Although countries around the world are committed to promoting the development and application of medical data and pay great attention to the protection of personal health information, the risk attributes of personal health information have rarely been mentioned before. This article first introduces the origin and development of medical big data, paving the way for the special risks faced by personal health information in this context. Then, through the introduction of concepts and characteristics, the content of personal health information is accurately defined. Next, according to a large number of personal health information security incidents, the new semantic scope of personal health information risk in the medical big data environment is analyzed, the necessity of personal health information risk regulation is emphasized, and the value conflicts that may occur in the process of personal health information risk regulation are clarified, laying the groundwork for the establishment of the risk decision-making procedure in the following article.

## 1. Introduction

The rapid development of the Internet and the emergence of emerging technologies such as cloud storage and cloud computing have made all kinds of data in modern society grow explosively, and the concept of big data has emerged and risen in this process. Nowadays, big data has shown great value and is widely used in various fields of economy and society [1]. The development of medical big data is the deep integration of big data and the medical industry, which is of great significance for clinical treatment, infectious disease prevention, drug research and development, etc. In this process, personal health information increasingly appears in all aspects of the medical-related field, and the in-depth analysis of data and the sharing of information between institutions continue to explore the scientific research and commercial value of personal health information, but also make the risk of personal health information being leaked more and more. On the other hand, personal health information is placed in the context of big data, and the huge scale of data makes the harm in the event of a leak accident that is unmatched in the past.

In the face of the threat of a risk society, the risk prevention mechanism of modern society does not seem to be fully prepared. Although each country and region have adopted the necessary protection measures for personal health information in different ways, due to the particularity and sensitivity of the content, the response to the risk of personal health information is higher than that of general information. At present, regulatory theories and schemes oriented to modern risks are mainly concentrated in the fields of nuclear safety, environmental safety, and food safety, while the risk attributes of personal health information are almost not mentioned. But in fact, the emergence of medical big data has rapidly magnified the risk of personal health information to a level that cannot be ignored. Therefore, how to take effective measures to control the risk of personal health information in the big data environment will be a problem we have to think about [2].

## 2. Personal Health Information under Medical Data

The concept of big data and related technologies was born during the explosive growth of the Internet industry, dating back to around 2000. Its real attention stems from its outstanding performance in the economic field, with the release of research on the big data-driven economy by well-known research institutions such as McKinsey and the World Economic Forum in 2011, and a big data boom has been set off worldwide. Big data has become a hot topic in recent years, accurately grasping the characteristics of big data 4 V: namely, volatile (scale), variety (diversity), velocity (real time), and value (value) are the keys to understanding big data, as shown in Figure 1.

At present, the emerging technology industry represented by big data not only is an important driving force for China's economic development, but also profoundly changes people's way of life. Under the dual role of policy support and social needs, China's big data industry has also shown a healthy and rapid development trend in recent years. It is estimated that the scale of China's big data core industry will reach 58.6 billion yuan in 2020 [3]. The changes that big data has made to people's lives are reflected not only in the huge growth of economic scale, but also in all aspects of people's lives. The deep integration of big data with the government and other industries is an important driving force for the formation of innovative development, and it is also the most direct embodiment of improving people's lives. In the “Internet+” model, big data is widely used, “Internet + government affairs,” “Internet + education,” “Internet + culture,” “Internet + transportation,” etc., using public management, education, culture, transportation, and other fields of big data to develop a variety of convenient applications and platforms, greatly facilitating the daily life of the people, but also greatly improving business efficiency. “Internet + medical” is produced in this context, and the application of big data in the medical field, for disease treatment, infectious disease prevention, medical technology development, and hospital management, has far-reaching significance. Personal health information is an important part of medical big data, and its value can be fully explored to improve the level of medical and health services and other significance, the development of medical big data technology is also moving in this direction to a large extent, but at the same time, new technology also brings new risks to personal health information security. In order to achieve effective risk management, it is important to understand the risk specificity of medical big data and personal health information [4–6], as shown in Figure 2.

### 2.1. The Definition and Connotation of Personal Health Information

Personal health information is an important part of personal information, and clarifying the concept of personal information helps to correctly define personal health information. Although there are differences in the definition of personal information and the enumeration of specific types of personal information in different laws and regulations in China, they all recognize the “identification theory” of personal information; that is, the main feature of personal information is that it can identify specific individuals, and the Cybersecurity Law defines personal information as “All kinds of information recorded electronically or otherwise that can be used alone or in combination with other information to identify a natural person personally.”

Privacy and personal medical information protection correspond to private and sensitive information, respectively. The difference between the two is mainly reflected in the fact that private information and sensitive information belong to different types of protection, which correspond to different types and methods of protection of civil rights and interests, and have different emphases [7]. In addition, the distinction between sensitive and nonsensitive information stems from the fact that the behavior of information processors is oriented to different objects, and the Personal Information Protection Law regulates from the perspective of personal information processing, focusing on the interpretation of the dimensions of individual information protection.

Broken down into the medical field, medical activities will involve a large amount of personal health information. However, China's laws are less related to the protection of personal health information, and the concept of personal health information has not been uniformly identified. Article 3 of the Measures for the Administration of Population Health Information (Trial Implementation) stipulates that personal health information is the basic population information and medical and health service information generated in various types of medical and health service establishments [8]. The “Information Security Technology Personal Information Security Specification” stipulates that personal health and physiological information only refers to various types of medical records and other information related to personal physical health conditions generated by personal illness and treatment. There is also no consensus on the definition and connotation of personal health information. Some scholars believe that “personal health medical information mainly refers to personal body characteristics, health status, interpersonal contact, genetics, medical history, and medical records involved in the process of physical examination, diagnosis, treatment, disease control, medical research process, etc.,” and some scholars believe that “personal medical information not only includes the physical or mental health of the information subject, and information such as medical conditions also includes basic personal information and personal economic information related to medical treatment.” It can be seen that the main controversy in the definition of personal health information in China's academic and legislative circles is whether personal health information is limited to information related to personal physiological and mental health conditions, and whether it can also contain basic personal information and economic information related to medical treatment.

Figure 3 shows the whole process of residents seeking medical treatment. China's personal health information is mainly generated in medical and health activities, so by analyzing the information generated in the process of personal medical treatment, we can better define the definition and connotation of personal health information. During the process of personal medical treatment, the doctor must provide the doctor with basic personal information such as his name, gender, and contact information, as well as relevant health information such as symptoms, family genetic history, and past medical history. In the process of diagnosis and treatment, the doctor produces the patient's symptom records, CT, and other examination records, and surgical conditions and other diagnosis and treatment information. It can be seen that the information generated by individuals receiving medical services is composed of two parts: personal identity information and diagnosis and treatment information; the former is the general personal information that can identify a specific natural person, and the latter is the information related to medical behavior involving the physical and mental health of the individual. In order to distinguish between the protection of personal health information and general personal information, the author believes that personal health information refers to information related to an individual's physical and mental health conditions generated in medical activities such as physical examination, diagnosis, and treatment, and can be identified individually or in combination with other information. Its content mainly includes basic health information that can help correct diagnosis and treatment, such as clinical symptoms, family medical history, drug allergy history, and past medical history, and health information generated in the process of medical services, such as examination results, surgical records, and anesthesia records [9–11].

### 2.2. Identification of Personal Health Information and Medical Privacy

When it comes to the protection of personal health information, it is easy to link it with patient privacy, and there are many scholars in the relevant literature who equate patient privacy with personal health information protection. But in fact, protected personal health information and patient privacy are two different concepts. Privacy and personal medical information protection correspond to private and sensitive information, respectively. The difference between the two is mainly reflected in the fact that private information and sensitive information belong to different types of protection, which correspond to different types and methods of protection of civil rights and interests, and have different emphases. In addition, the distinction between sensitive and nonsensitive information stems from the fact that the behavior of information processors is oriented to different objects, and the Personal Information Protection Law regulates from the perspective of personal information processing, focusing on the interpretation of the dimensions of individual information protection, as shown in Figure 4.

1. The extensions of the two intersect with each other. China's legislation does not clearly define the connotation of privacy, but from the analysis of the semantic interpretation of privacy and the relevant legislative provisions, the academic circles generally believe that privacy generally refers to the private secrets of personal private life tranquility or private life information that individuals do not want to disclose or are inconvenient to be known by others [12]. (2) Medical privacy emphasizes privacy and nondisclosure, including the patient's personal body privacy, the patient's medical information privacy, and the patient's personal space privacy. The important feature of personal health information lies in the identity of the subject; that is, others can identify a subject through this health information. Some health information that can identify the information subject himself or herself that is not disclosed is health privacy, but personal health information includes not only health privacy information that does not want others to know, but also information that has been disclosed.
2. Whether or not there is a property interest is different. Medical privacy contains personal interests, closely related to the reputation and dignity of individuals, and infringement of personal privacy will often cause personal life tranquility destruction and personal spiritual pain, and will not cause damage to personal property interests. Although personal health information also points to the personal dignity and interests of the information subject, it also contains property value. In the information age, various institutions and organizations have gradually tapped the economic value of personal health information. Personal health information can help organizations achieve business activities such as customer base profiling, market condition surveys, and strategy development. At the same time, after processing, health information itself becomes a data product that can be traded.
3. It is different from the relevance of the public interest. Privacy is information that private individuals do not want others to know or that is inconvenient for others to know, and it is generally considered that the domain belonging to the self is not closely related to the public interest. Unlike privacy, personal health information is closely related to the public interest, and personal health information itself has public welfare value. Especially in the prevention and treatment of the epidemic and medical research, the collection and processing of personal health information can help the progress and development of medicine [13].

### 2.3. The Legitimacy of Special Protection of Personal Health Information

#### 2.3.1. The Particularity of Personal Health Information Itself

In addition to the common characteristics of general personal information such as identifiability, personal health information has its particularity due to the high professionalism and particularity of medical activities, which is mainly reflected in the following aspects:

1. Personal health information is sensitive and carries higher personality interests. Although there is no consensus in the academic circles on the legal attributes of personal information, it is recognized that personal information carries personality interests. Through the collection of personal information, the information subject's information personality is formed, ensuring the consistency and authenticity of personal information and the true self, and the information subject's control over its information, which is related to the personal dignity and personality autonomy of the information subject, and carries the most basic personality rights and interests that the information subject should enjoy. (2) Personal health information involves private and sensitive information such as personal health status, which is more closely related to personal dignity, and once it suffers damage, the damage to the information subject is more lethal. Due to the professionalism of medical service activities, personal health information is mostly composed of various medical terms and professional terms, such as hepatitis B antibodies and antigen detection indicators. It is difficult for nonmedical professionals to correctly understand the actual meaning of various types of information, and it is easy to misunderstand the information subject [14]. Therefore, the improper disclosure of personal health information or other violations can easily cause the social evaluation of individuals by the outside world to decline, so that individuals suffer discrimination in social life such as employment and insurance, and even cause great psychological pressure to individuals [15]. For example, although the law stipulates that except for certain specific occupations, employment may not be refused on the grounds of having hepatitis B, there have been many cases of discrimination against the employment of hepatitis B virus carriers in China.
2. Vulnerability of personal health information. First, healthcare organizations are able to quickly and accurately collect patients' personal health information. Personal health information is mostly generated in medical behavior, and patients will consciously take the initiative to medical staff out of their emphasis on personal life and health and trust in medical staff Disclose a large amount of personal health information [16]. The medical activities are highly professional and complex, and patients are unable to judge on their own whether the collection of personal health information in the process of medical service provision exceeds the necessary limits due to the lack of medical knowledge. In the general network information collection, consumers can choose not to disclose their personal information, but patients lack selectivity in the process of personal health information collection. Patients have the obligation to cooperate with medical institutions in the process of medical treatment and provide comprehensive and accurate personal health-related information. Second, the subjects of personal health information that can be contacted are diversified and complicated. Medical services involve multiple business process nodes such as “registration, consultation, inspection, examination, and treatment,” and the staff of each node, such as doctors, nurses, and medical administrators, may have access to the patient's health information [13]. (1) The widespread use of electronic medical records has changed the path of dissemination and control of medical information, enabling more unauthorized institutions or individuals to easily access personal health information. The openness and sharing of the Internet enable multiple users to use the same kind of electronic medical records at the same time, and personnel in different regions can also remotely access electronic medical records. (2) Patient health information can break through the limitations of space to use, store, circulate, and transmit between multiple departments. For example, in 2017, Chongqing completed the interconnection of electronic medical records of various medical institutions in the county and realized the sharing of electronic medical records across medical institutions. The open nature of the network significantly expands the range of subjects that can be reached, not only within the medical institution but also to the third-party commercial institutions on which the electronic medical record is established. Finally, patients have poor awareness of the protection of their personal health information and cannot choose to delete their personal health information. The protection of personal health information in China's laws mainly depends on the provisions on the confidentiality obligations of medical institutions, and patients only pay attention to the prevention and treatment of their own diseases and pay little attention to the subsequent use and storage of personal health information, giving criminals the opportunity to take advantage. In the general personal information, the information subject may request the correction or deletion of personal information. In medical activities, the law clearly stipulates that medical institutions have the obligation to keep patients' medical records, and medical institutions must properly keep patients' medical records within the statutory time, so the information subject requires medical institutions to delete the records of personal health information subject to time restrictions. As a result, personal health information is more vulnerable to infringement than general personal information.
3. The comprehensive utilization value of personal health information is high. Employers, insurance companies, drug manufacturers, and medical researchers all want access to a wealth of personal health information for analysis. (3) For relevant institutions engaged in the health industry, the analysis and utilization of personal health information can generate great commercial value. For example, pharmaceutical manufacturers can tap market demand, develop new products, and carry out precision marketing by analyzing personal health information; medical service institutions can form a personal health portrait of the information subject through a comprehensive analysis of personal health information and provide customers with personalized health service programs [13]. (4) In addition to being used for the treatment of individual patients, personal health information plays a major role in the prevention and treatment of epidemics, medical research and education, and the allocation of medical resources. (1) If an epidemic or infectious disease breaks out, it can be developed by collecting patient health information for epidemiological statistical analysis. Without sufficient accurate and comprehensive information on the causes and routes of transmission, the identification of disease outbreaks may be delayed to an extent that is difficult to control [17]. Health facilities can use personal health information to analyze population health trends, compare the cost and quality of care, and compare and evaluate treatment outcomes. Through the tracking and analysis of personal health information, medical research institutions can help researchers understand the natural process of diseases or the complex relationship between different diseases, promote the development of national medical technology level and quality, and provide the possibility of curing difficult medical records. (2) The state can obtain a complete national health information database after collecting and processing national health information, according to a large amount of information in the information database, the state can carry out disease prevention and rational allocation of medical resources, and personal health information can become a national strategic resource. Therefore, personal health information has both commercial value and public welfare value.

#### 2.3.2. The Inevitable Requirements of the Information Age

Technical issues are the primary problem facing the development of medical big data, which directly affects whether medical big data can develop rapidly and effectively, and whether it can play a key role in the construction of digital health. Compared with the backward level of technology that may bring about the low efficiency of medical big data applications, the ethical problems faced by medical big data may be more severe. In the era of medical big data, patients' personal health information is widely present in mobile apps and the Internet. The massive, interactive, shared, dynamic, and other characteristics of medical big data determine that compared with the traditional medical data storage and application methods, the risk of personal health information leakage is undoubtedly significantly increased in the era of medical big data.

#### 2.3.3. Necessary Conditions for the Cross-Border Flow of Personal Health Information

In the information age, the cross-border flow of personal health information has become the norm, and the personal information protection law generally has extraterritorial effects. Judging from the personal information protection laws enacted by many countries and regions, they all try to distinguish between the protection of sensitive information and general personal information. Although the sensitivity of citizens of various countries to different information is not consistent based on the different historical and cultural backgrounds of various countries, it is stipulated that personal health information is sensitive information and personal health information is strictly protected. For example, in 1981, the European Council promulgated the Agreement on the Protection of Individuals concerning the Automated Processing of Personal Data, which for the first time clearly defined sensitive personal information and made special provisions for the automated processing of such information. Since then, in the process of data legislation in the European Union, the types of special data have been clarified and the collection and processing of such data have been strictly restricted. Legislation on the protection of sensitive personal information in the USA is fragmented, and specific information protection laws are enacted in certain industries. For personal health information in the medical industry, the USA has specially enacted the HIPPA Act to protect personal health information [18].

Personal health information in the information age is not only related to the personal interests of information subjects, but also becomes an emerging strategic resource of the country. At present, in the international information exchange activities, many countries outside the region have formulated strict requirements and standards for the protection of personal health information, and if the protection of health information in China does not meet the standards formulated by countries outside the region, it will restrict the exchange of information between China and them, and even refuse China's information exchange activities. Therefore, in the face of the universality of special protection of personal health information outside the region, if special protection is not given to personal health information, it will lead to the “double standard” of personal health information protection at home and abroad, and China will not be able to carry out equal health information exchange and trade with the European Union, the USA, and other countries. The strict protection of personal health information outside the region makes it impossible for relevant institutions in China to obtain the health information of foreign citizens. On the contrary, China's loose protection of personal health information allows institutions outside the country to easily obtain personal health information of Chinese citizens and then use large quantities of health information for commercial or research activities, which will threaten China's economic and social development and even endanger national security. To this end, China has tried to protect personal information based on the sensitivity of information. For example, China's criminal law first focused on the protection of personal information, and as early as 2009, the serious violation of personal information was classified as a criminal act. With the refinement of the determination of the crime of infringing personal information, China adopts the criteria of “five hundred articles” or more for the determination of “serious circumstances” of infringement of personal health information, compared with general personal information. More than 5,000″ criminalization standards, China's criminal field has taken stronger protective measures for personal health information than ordinary information. Regrettably, the protection of personal health information in the field of private law in our country is still weak [19].

## 3. The Risks Faced by Personal Health Information in the Big Data Environment

### 3.1. Analysis of the Types of Infringement of Personal Health Information

In the process of large-scale medical informatization reform, the important use value of personal health information has been highlighted, and the types of personal health information infringements have been varied. According to the circulation process of personal health information, the specific types of violations are divided into four aspects: improper collection of personal health information, improper disclosure of personal health information, improper use of personal health information, and improper preservation of personal health information.

#### 3.1.1. Improper Collection of Personal Health Information

Illegal collection and excessive collection of personal health information are improper collection of personal health information. Illegal collection refers to the collection of health information by others without a lawful basis for information collectors and the improper collection of health information. For example, in the case of “Dispute over the Privacy Rights of Zhang X, Zhang X A, etc., with Suiping County People's Hospital and Wei X X,” the defendant illegally collected the patient's medical records from other institutions without the consent of the patient and without legal procedures, for the needs of his litigation interests, and presented it in another litigation trial. Excessive collection refers to the collection of personal health information beyond the specific purpose of collection and the collection of health information unrelated to the specific purpose of collection.

The subjects of personal health information collection include healthcare providers and nonmedical service providers. For medical service providers, the collection of personal health information is a prerequisite for the development of medical and health activities, and the basic information and health and physiological conditions of individuals are the basic information necessary for medical activities. However, China's laws lack provisions on the scope, subjects, and procedures for collecting personal health information. In reality, various medical service institutions often collect according to the actual needs of their own work, and a large amount of information is collected repeatedly. At the same time, patients lack the ability to identify the scope of personal health information collection and self-protection awareness, and medical institutions such as hospitals often over-collect personal health information for utilitarian purposes. For nonhealthcare providers, the commercial value of personal health information often attracts them to excessively collect or even illegally collect personal health information out of the needs of their own interests, causing harm to the information subject, as shown in Figure 5.

#### 3.1.2. Improper Disclosure of Personal Health Information

Personal health information controllers disclosing or providing personal health information to other institutions or individuals without the explicit consent of the information subject or without other legitimate reasons are an improper disclosure of personal health information. In practice, there are many incidents of improper public disclosure of personal health information. For example, in the case of Lü Weiwei, Tang Baohua, and others in a dispute over the right to reputation with Hubei Radio and Television Station and Wuhan Mental Health Centre, the hospital provided the patient's medical record information to the TV station without the consent of the guardian of the mentally ill patient, and the TV station made it public, bringing great mental pressure to the patient.

Both traditional medical ethics and laws clarify the obligation of medical service providers to keep personal health information confidential, and personal health information shall not be disclosed without the consent of patients. The illegality of improper disclosure of personal health information is mainly manifested in the infringement of the right of information subjects to independently decide whether their health information can be known by others and under what circumstances. Improper disclosure will make the personal health information of the information subject known to the unspecified person in society, which is very likely to affect the personal dignity and freedom of the information subject. Judgments on improper disclosure shall be based on whether there is a lawful basis for disclosure.

#### 3.1.3. Improper Use of Personal Health Information

Improper use of personal health information includes the use of personal health information in violation of the scope of laws or agreements, the unauthorized use of personal health information of information subjects, the illegal use of personal health information for the purpose of information collection, and the illegal transaction of personal health information. For example, the medical staff of a hospital in Anshan City took advantage of their positions to sell the personal information of patients in the hospital to the milk powder sales personnel, and after investigation by the public security organs, the personnel sold more than 20,000 pieces of personal information of patients. A hospital in Rizhao, Shandong Province, introduced a set of tumor treatment equipment, in order to better create economic benefits, the use of television, newspapers, and other media without authorization to publicize and report the medical information of patient Wang's use of the equipment, which seriously affected Wang's normal life and caused Wang's mental pain.

The use of personal health information shall be controlled by the information subject, but once the personal health information is collected by the information collector, the individual's ability to control the health information is weakened, and the information collection controller can secretly complete the processing and use of personal health information. Once the information controller illegally or excessively uses personal health information, the damage to the information subject's control over personal health information is often accompanied by damage to the property interests of the information subject and the intrusion of the tranquility of private life, as shown in Figure 6.

#### 3.1.4. Improper Storage of Personal Health Information

After the collection of personal health information, it is also necessary to save it legally, and the act of deleting or modifying personal health information in violation of regulations, or not keeping personal health information in accordance with regulations, causing information leakage is improper preservation of personal health information. With the advent of the era of medical informatization, electronic health information is more likely to be tampered with, the information asymmetry between information subjects and information collectors is becoming more and more serious, and it is often difficult for individuals to detect the deletion and modification of personal health information. For example, in the case of the privacy dispute between Cun Lili and Beijing Anorectal Hospital, the defendant's medical record data management was not strict, resulting in the disclosure of the plaintiff's medical records, and the illegal merchants published the plaintiff's medical records online without the consent of the plaintiff and made them into CDs for sale, causing great mental damage to the plaintiff. A patient hospitalized in a hospital in Jiangxi Province had a dispute with the hospital due to a medical accident, the hospital falsified its medical records in order to win the lawsuit, resulting in obvious alteration of medical records, and the handwriting was also different in many places.

As can be seen from the above-mentioned cases, violations of improper preservation include both positive actions and negative omissions. The unlawfulness of improper preservation of personal health information is manifested in the damage to the completeness, accuracy, and safety of the information subject's personal health information. The complete accuracy and safety of personal health information are related to the personality rights and interests of the information subject. Maslow pointed out that “the integrity and authenticity of personality identification are the basic conditions for the subject to be respected by others.” The accuracy and completeness of personal health information can ensure that the personal health profile of the information subject is not distorted, and the information subject can live with dignity.

### 3.2. The Current Situation of Personal Health Information Protection in China

At this stage, my country's personal information protection law is still in the drafting stage, and the legal provisions on personal health information protection are limited and scattered in the legal system of various departments, as shown in Table 1. At present, there are two modes of privacy protection mode and behavior regulation mode for the protection of personal health information in my country.

#### 3.2.1. Privacy Model for Personal Health Information Protection

Privacy, especially patient privacy, is closely related to personal health information, so for a long time, China has relied on privacy to protect personal health information. As early as 1998, the Interpretation on Several Issues Concerning the Trial of Reputation Cases stipulated that medical personnel disclosed the condition of patients with sensitive diseases such as gonorrhea and syphilis without authorization and caused damage to the patient's reputation infringed on the patient's right to reputation, and medical privacy was included in the scope of protection of the right to reputation. With the promulgation of the Interpretation on Compensation for Moral Damages [2001] No. 7, privacy and reputation exist independently. The Law on Practicing Physicians, the Law on the Prevention and Control of Infectious Diseases, the Regulations on the Management of Medical Records of Medical Institutions, the Regulations on Nurses, and other health legislation stipulate the confidentiality obligations of medical institutions and medical personnel to the privacy of patients and stipulate that those who violate the confidentiality obligations shall bear administrative responsibility or even criminal liability. With the promulgation of the Tort Liability Law, the right to privacy began to emerge as an independent civil right. Article 62 of the Tort Liability Law stipulates that the privacy of the victim shall be exposed or disclosed. From the above legislative practice, it can be seen that China's privacy rights have experienced from “relying on the protection of the right to reputation” to “privacy interests” to “privacy rights.” The evolution of the process. Article 12 of the 2014 Provisions on Several Issues Concerning the Application of Law in the Trial of Civil Dispute Cases Involving the Use of Information Networks to Infringe Personal Rights and Interests clearly stipulates that the medical record data of natural persons belong to personal privacy, and the protection of personal health information with privacy rights is gradually developed.

#### 3.2.2. Code of Conduct for the Protection of Personal Health Information

The General Provisions of the Civil Law promulgated in 2017 set personal information independent of privacy protection and determined that the interests of personal information became legal interests that could be independently protected. However, the General Provisions do not set the right to personal information for information subjects, but protect personal information by regulating the behavior of information collection controllers. The 92nd Law on Basic Medical Care and Health Promotion, promulgated in December 2019, stipulates that “the state protects citizens' personal health information and ensures the security of citizens' personal health information.” Citizens' personal health information must not be illegally collected, used, processed, or transmitted by any organization or individual, and must not illegally buy, sell, provide, or disclose citizens' personal health information. “As the basic law in the field of medical and health care, it declares the protection of personal health information, is highly in line with the provisions of the General Provisions of the Civil Law on the protection of personal information, and limits the behavior of the controller of information collection in the form of behavior constraints.” Article 111 of the General Provisions of the Civil Law and Article 92 of the Basic Medical Care and Health Promotion Law define the code of conduct for the three stages of collecting, using, and possessing personal health information. However, the above-mentioned provisions on the determination of “legal” and “illegal” need to be transferred to the relevant provisions of the Cybersecurity Law and the Measures for the Administration of Population Health Information.

Stage of collection and use of personal health information: Article 8 of the Measures for the Administration of Population Health Information stipulates that the collection and use of personal health information must comply with the principle of “minimum adequacy.” Article 41 of the Cybersecurity Law stipulates that the collection of personal information must meet the principles of legitimacy and necessity and informed consent. Among them, the principle of “minimum sufficiency” can be absorbed in terms of effect into the principle of legitimacy and necessity. Specifically, the “principle of propriety and necessity” requires that users of information collection only collect personal health information that is necessary for business applications. The principle of “informed consent” requires that the purpose, method, and scope of personal health information collection must be open and transparent and must obtain the consent of users.

Personal health information holding stage: The information collection controller has the obligation to ensure the safety of personal health information. The Cybersecurity Law and the Measures for the Administration of Population Health Information stipulate that health information collectors should establish an information confidentiality system and take technical protection measures, remedial measures for information leakage, and notification rules.

The code of conduct model can provide a certain basis for judging the illegality of personal health information infringement in judicial practice and, to a certain extent, make up for the lack of discretion of judges' illegality judgments. The behavior guidance of information collectors and users in the whole process of health information circulation protects personal health information from the source and makes up for the lack of protection at the end of privacy.

### 3.3. Insufficient Protection of Personal Health Information in China

#### 3.3.1. Lack of Legislation on the Specificity of Personal Information

For a long time, Chinese scholars have paid attention to the protection of personal information and formulated several drafts of the Personal Information Protection Law (Expert Suggestion Draft). However, China's Personal Information Protection Law has not yet been promulgated, the special legislation for personal information protection is lacking, and the definition of personal information concepts and connotations is vague, not to mention the definition of personal health information. Judging from the legal norms for the protection of personal health information, the overall distribution is scattered and the legislation is trivial. Judging from the legislative level involving laws on the protection of personal health information, most of them are distributed in medical regulations with lower effectiveness levels, and most of them are administrative regulations or departmental rules. From the content of the legal provisions, many legal provisions only macroscopically emphasize the confidentiality obligations of medical institutions and medical personnel to personal health information, but for how to protect personal health information, the responsibility for infringing personal health information and other specific supporting systems are not perfect, so the current legal provisions are mostly the principle of protecting personal health information, which is poorly operable, which is embodied in the following: on the one hand, the law cannot reasonably guide the behavior of information collection controllers to collect and process personal health information. On the other hand, the rights and interests of information subjects for personal health information are not clear, and when the personal health information of information subjects is infringed, the information subjects cannot effectively safeguard their rights.

#### 3.3.2. The Scope of Legal Benefit Protection for Health Information Subjects Is Narrow

In the information age, the protection needs of information subjects for personal health information have changed from passive defense to active control and utilization. The scope of legal interest protection of information subjects shall include all rights and interests related to information control and utilization, such as the knowledge, modification, and inquiry of information.

Rights protection legislation can directly define the scope of legal interests of information subjects. China has not enacted legislation to confirm the right to personal information, but has used privacy rights to protect the rights and interests of information subjects. As a passive defensive right, the core right of privacy lies in keeping secrets for the subject's private affairs, eliminating illegal intrusion, mainly in resisting intrusion and disclosure, dominating personal secrets and private living space, and excluding the intervention of others as the content of rights and interests. For information subjects in the information age, the legal benefits that information subjects should enjoy for personal health information are not only limited to passive defenses to avoid interference by others, but also reflected in the information subject's active control and use of personal health information. Therefore, the simple privacy protection model limits the scope of legal protection of information subjects.

The code of conduct legislation restricts the scope of information subjects' rights and interests by restricting the conduct of the actor. The General Provisions of the Civil Code and the Law on Basic Health Care and Health Promotion provide a negative list of the conduct of information collectors, but the negative list is closed and cannot comprehensively enumerate all the ways of conduct. It can be seen from the interpretation of the legal text that acts that do not belong to the negative list should be attributed to the freedom of conduct of the information collectors and users, so the normative legislation significantly narrows the scope of legal interest protection for information subjects.

#### 3.3.3. The Protection of Personal Health Information and General Personal Information Has Not Been Realized

Personal health information is sensitive personal information, and special protection of personal health information is legitimate. At present, China's private law adopts a single behavior regulation for the collection, processing, and preservation of personal information, and information collection and processors in all aspects of information circulation need to comply with certain legal rules, mainly including the principle of legitimacy and necessity, the principle of informed consent, and the principle of security guarantees. However, from the perspective of the comparison between the general personal information and the personal health information protection rules, the law does not make special provisions on the principles for the collection and processing of personal health information, and there is no difference between the collection and processing of personal health information by the information collection and processing personnel and the general personal information, and the special protection of personal health information cannot be realized.

### 3.4. Lack of Civil Remedies for Health Information

From the perspective of the relief mechanism for infringement of personal health information, there is a legislative concept of emphasizing “criminal punishment and administrative management” over “civil relief,” and health legislation tends to administrative and criminal remedies, stipulating administrative and criminal liability for infringement of personal health information, but lacking provisions on civil attribution and compensation. The personal interests and property interests suffered by the information subjects themselves cannot be compensated accordingly. For offenders, the lack of civil compensation provisions reduces the cost of violating the law by the perpetrators, further causing the rampant infringement of personal health information. Although the General Provisions of the Civil Law make it clear that personal information is protected, it does not make specific provisions on civil liability for acts of infringement of personal information. Judging from the judicial practice of personal information protection in China, when the health information of the information subject is infringed, the court still adopts the privacy right approach to remedy the rights and interests of the information subject.

The Tort Liability Law adopts enumerative provisions on the way of infringement of patient privacy and only stipulates two kinds of infringements: “leakage” and “disclosure of medical record information without consent.” From the above analysis of the types of personal health information infringement, it can be seen that the infringement of personal health information in the information age not only is limited to improper disclosure and leakage, but also appears in a large number of improper collection, use, preservation, etc. All aspects of the circulation of personal health information may have various types of infringements. Therefore, the limited nature of the provisions on infringement is difficult to achieve effective remedies for information subjects. The Tort Liability Law lists the circumstances in which the principle of presumption of attribution of fault is applied to the infringement of medical damages, but does not include situations in which medical institutions and medical personnel infringe on the privacy of patients. According to the regulations, the principle of attribution of fault is applied to tort liability for tort liability that does not clearly stipulate the application of the principle of presumption of fault, and the information subject whose health information has been infringed provides evidence to prove that the medical institution and medical personnel are at fault. However, the information of the information subject and the information collection controller is asymmetrical, the information subject is difficult to prove, and it is difficult to determine the infringer, the specific infringement, and the loss of the information subject, especially the economic loss. As mentioned above, in the context of medical informatization, the number of organizations and personnel that can access personal health information is increasing, the channels and channels of health information infringement are diverse, and it is difficult for the victim information subject to determine the specific infringer. The development of medical informatization has made the infringement of personal health information hidden, and it is often difficult for information subjects to detect the infringement. Therefore, it is significantly more difficult to protect the rights of information subjects when their personal health information is infringed.

At present, the protection of personal health and medical information in China has not yet formed a systematic legal norm, but only fragmented provisions in the provisions of laws and regulations, although the health and medical management departments to develop internal information security management norms, but generally not mandatory, data collection, storage and utilization more rely on self-discipline management. How to punish the improper handling of personal health and medical information is not particularly specific, and most of them are only relatively rough provisions in the Civil Code, the Public Security Administration Punishment Law, the Cybersecurity Law, the Basic Medical Care and Health Promotion Law, the Criminal Law, and other laws and regulations.

## 4. Improve China's Personal Health Information Protection Mechanisms

### 4.1. Enact a Unified Personal Information Protection Law

In view of the scattered legal provisions on the protection of personal information in China, most of which are legislative status quo stipulated in principle, it is impossible to effectively protect the personal health information of information subjects, and the special legislation on personal information protection is urgent. From the perspective of legislative models, the EU and the USA are typical representatives of unified legislation and decentralized legislation. The European Union regulates uniform legislation on the collection, processing, and retention of personal information by controllers of information collection. The unified legislative model can apply relatively consistent standards to protect personal information, avoid conflicts of legal application between different laws, and provide strict protection for personal information. However, the value orientation of information protection and circulation in different industries may be different, and the one-size-fits-all legislative model may not be able to meet the requirements of information circulation in some industries. The decentralized legislative model of the USA can combine the characteristics of personal information in different industries for special legislation, which helps to protect sensitive personal information in particular and promote the circulation and sharing of general personal information. However, the decentralized legislative model will increase the cost of national legislation, and there will be overlaps between multiple laws, resulting in confusion and application of legal provisions.

As a civil law country, China has a more realistic basis for formulating a unified written law in China. In 2006, Zhou Hanhua formulated China's first “Personal Information Protection Law (Expert Proposal Draft),” and since then, many proposals formulated by Chinese scholars have generally adopted a unified legislative model to protect personal information. Among them, the “Personal Information Protection Law (Expert Proposal Draft)” formulated by Zhang Xinbao and Ge Xin, under the premise of adopting a unified legislative model, is based on the concept of “two-end strengthening and tripartite balance,” and legislation strengthens the protection of personal sensitive information and the use of personal general information. The Draft Recommendation stipulates that information subjects have the right to inquire and correct personal information, and stipulates the principle of “special protection of sensitive personal information.” For the protection of sensitive information such as personal health information, the Draft Recommendation stipulates that information controllers shall take measures to specifically protect the sensitive information of information subjects, must not collect sensitive information, and specially remind information subjects when collecting sensitive information.

In the absence of China's personal information protection legislation, the formulation of a unified “Personal Information Protection Law” is more in line with China's legislative tradition and reality. For more sensitive personal health information, special rules may be formulated in the Personal Information Protection Law for special protection on the basis of Zhang Xinbao and Ge Xin's draft proposals. Under the framework of the Personal Information Protection Law, specific rules for the protection of personal health information may be gradually formulated, and comprehensive protection may be implemented for the circulation process such as the collection, processing, and preservation of personal health information.

### 4.2. Expand the Scope of Legal Interest Protection for Information Subjects

From the above analysis, it can be seen that the establishment of the right to personal health information can expand the scope of legal protection of information subjects and realize the control of personal health information by information subjects. The right to personal health information refers to the right of individuals to control and exclude infringement by others from the data formed by their own health status in accordance with the law. Clarify the right to personal health information. The subject of the right to personal health information directly points to the natural person, the object is the identifiable personal health information, and the content of the civil right determines the scope of legal interest protection of the right subject. Therefore, on the basis of clarifying the subject and object of the individual's right to health, further elaborating the content of their rights is conducive to clarifying the legitimate rights and interests enjoyed by the subject of health information and laying the foundation for the protection of personal health information.

#### 4.2.1. The Right to Know Personal Health Information

The right to know personal health information is the basic right of the information subject, which means that the information subject has the right to know all information related to the collection, processing, and preservation of personal health information, including the identity of the health information collection controller, the purpose of collection and use, the scope of collection, the processing situation, and the information security protection measures.

#### 4.2.2. Control of Personal Health Information

Personal health information control means that the information subject has the final right to make decisions on personal health information. Specifically, it includes the right to consent, the right to rectification, the right to erasure, and the right to block.

The right to consent is the most important right to reflect the information subject's control of personal health information, and through the consent of the information subject, it is decided whether others can collect, use, and disclose personal health information. At present, there are two main ways to realize the right of consent of individuals in the world: one is the opt-in mechanism; that is, only with the consent of the information subject, the information collection and user can collect and use personal health information, and through reasonable notification procedures, the information subject can withdraw its previous opinions at any time. The second is the opt-out mechanism. Personal health information may be collected and used as long as the individual does not explicitly refuse, but the information subject has the right to request the withdrawal of consent at any time. The former focuses on the explicit consent of personal health information collection and processing, which is conducive to safeguarding the legitimate rights and interests of information subjects. The latter constructs an implicit consent rule for the collection and processing of personal health information, which ensures the circulation of personal health, but is not conducive to the protection of the rights and interests of information subjects. Personal health information is more closely related to personal dignity and freedom, so out of the need to protect the personal interests of information subjects, it is more appropriate to adopt a selective entry mechanism.

The right to rectification refers to the right of the information subject to request the information processor to correct or supplement the health information in the event that it finds that its personal health information is incorrect and incomplete or other quality defects. In the era of big data, massive personal information constructs the possibility of data portraits, and “data people” appear in large numbers. Through the collection and integration of personal health information, a personal health profile can be constructed. In the case of flawed health information quality, there will be distortions and inaccuracies in the portraits, leading to discrimination. Giving the information subject the right to correct can ensure that the personal health profile is infinitely close to the true personality of the information subject. However, it should be noted that the information subject does not have the right to correct all health information. Personal health information includes not only personal statement information and medical staff record information, but also information objectively formed by medical testing instruments such as imaging examinations. The quality defects of the former can be found to be corrected. The latter is not the subject of the right to correct personal health information, unless there is an artificial correction or a purely incorrect entry.

The right to erasure means that when certain conditions are met, the information subject has the right to request the health information controller to delete his personal health information in a timely manner, such as the information subject withdraws his consent, the specific purpose cannot be achieved, and the information is illegally processed. However, Article 29 of China's “Provisions on the Administration of Medical Records of Medical Institutions” stipulates the time for medical institutions to keep medical record data. Although the law does not explicitly stipulate the electronic medical record, the provisions of the paper medical record also apply to the electronic medical record. In the case that personal health information is under the control of traditional medical institutions, the right to delete the information subject is restricted, and patients cannot require medical institutions to destroy their medical record data within the statutory time. Under the “Internet + medical” model, many online consultation institutions, such as Doctor Lilac, have the functions of both network service providers and medical platforms, and the “Medical Record Management Regulations for Medical Institutions” cannot be applied to such medical service providers, so the information subjects have the right to request such institutions to delete personal health information.

The right to block means that the information subject has the right to request the personal health information processor to temporarily stop or restrict the processing of health information when certain conditions are met. The right of blockade is mainly applicable to emergencies that endanger the legitimate rights and interests of health information subjects, and to fix health information in order to prevent the occurrence of damage consequences or further expand the damage consequences in a timely manner. Article 16 of China's Regulations on the Handling of Medical Malpractice stipulates that patients and their close relatives shall enjoy the right to seal medical records after the occurrence of medical malpractice. Extended to the protection of health information, the right of information subjects to block has a legitimate basis in China.

#### 4.2.3. The Right to Decide on Personal Health Information

The right to decide on personal health information means that the information subject enjoys the right to use personal health information autonomously according to his own wishes; that is, he or she decides how to use this information, including when and where to share which health information, and enjoys the right to access and carry.

The right of access means that the information subject has the right to inquire about personal health information and the processing of the information and obtain a copy. Compared with the right to know, the right of access can better promote the information subject to grasp the processing and utilization of personal health information after collection and is an important right to promote the participation of information subjects in the circulation of information. In practice, personal health information is secretly processed and used without the knowledge of the information subject, and the granting of access rights can to a certain extent supervise the information processing behavior of the information collection controller and narrow the information asymmetry between the information subject and the information controller.

The right to portability means that the information subject has the right to transfer the personal health information he previously provided to the information collection controller to other information controllers or to require the original information collection controller to transfer his personal health information directly to another controller. The right to carry can strengthen the follow-up control of personal health information by information subjects, and at the same time, the right to carry can significantly avoid the phenomenon of repeated collection of patients in different medical institutions, thereby reducing the number of personal health information collected and protecting personal health information from the source.

#### 4.2.4. Right to Confidentiality of Personal Health Information

The right to confidentiality of personal health information refers to the right of information subjects to request that health information processors and controllers maintain the confidentiality of personal health information and must not illegally disclose their personal health information. Information subjects who wish to maintain the confidentiality of personal health information are core values of medicine and have been incorporated into the code of conduct for the medical profession. Medical institutions and medical personnel shall have the obligation to keep personal health information confidential based on medical ethics and laws and regulations, as shown in Figure 7.

The right to claim personal health information security is the right of the information subject to request the processor of personal health information to take necessary and reasonable protective measures, and also gives the information subject the right to file a lawsuit when the personal health information is infringed.

#### 4.2.5. Derogation of the Right to Personal Health Information

Information subjects have rights to personal health information, but the rights are not absolute, and in specific cases, the right to personal health information should make appropriate concessions and compromises. Personal health information carries the public interest and has important use value in medical research, epidemic prevention, and control. Therefore, the derogation of the right to personal health information is mainly reflected in the conflict with the public interest.

Taking epidemic prevention and control as an example, the outbreak of new coronary pneumonia in China has been controlled through national efforts. After the outbreak of the epidemic, the relevant departments carried out timely collection and analysis and utilization of the health information of new crown patients, and gradually updated the patient diagnosis and treatment plan, effectively saving the lives of more patients. Therefore, in the face of conflicts between the right to personal health information and the public interest, the protection of individual rights should be conceded to the use of public welfare. However, this does not mean that personal health information can be disclosed and used arbitrarily based on public welfare purposes, and out of the practical needs of the public interest, the disclosure and use of personal health information should comply with the principle of proportionality, the content should be really necessary, in line with the public welfare purpose, and the means of disclosure should be reasonable and appropriate.

### 4.3. Enhanced Protection of Personal Health Information

By establishing the form of protection for information subjects to enjoy personal health information rights, the scope of legal interest protection of information subjects can be directly and comprehensively defined. However, there are inherent structural defects in simply granting the right to personal health information to information subjects: (1) the rights of information subjects cannot be effectively exercised. Under the process of medical informatization, the collection and processing of personal health information can be completed covertly and quickly in the virtual space, and once it is separated from the information subject, the information subject basically loses the defector control and control over personal health information. Therefore, although the right to personal health information is given to the information subject, the right holder cannot actually control the personal information, and the rights are difficult to protect. In addition, the protection of rights requires clear remedies for rights, and the most important means of remedy lie in the determination and assumption of tort liability. The rights protection model cannot provide clear compliance guidelines and behavioral expectations for counterparts and cannot provide a clear basis for judging the illegality of tort law. (2) The scope of legal interest protection of personal health information and general personal information by information subjects: the difference is small, and it is difficult to achieve special protection of personal health information. By drawing on the special protection of health information by the European Union and the USA, it is found that both countries are proceeding from the code of conduct of information collection controllers, strictly limiting the collection and processing of personal health information by information collection controllers, so as to achieve the differential protection of personal health information and general personal information. Therefore, China should strictly limit the behavior of information collectors and users, and strengthen the protection of personal health information.

### 4.4. Improve Civil Remedy Mechanisms for the Protection of Personal Health Information

No remedy means no right. In order to ensure the realization of the right to personal health information, an effective infringement relief mechanism must be established. China's relevant legislation focuses on the administrative responsibility and criminal responsibility of the responsible subject and lacks a civil relief mechanism after the infringement of personal health information, which promotes the fluke psychology of health information collection and control, and there are a large number of infringements that do not yet constitute administrative punishment and criminal standards. Therefore, improving the civil relief mechanism can increase the illegal cost of information collection and processors, and at the same time promote the active protection of health information subjects.

#### 4.4.1. Improvement of Tort Liability for Infringement of Personal Health Information Rights

*(1) Determine the Principle of Attribution for Infringement of the Right to Personal Health Information*. The principle of fault liability is a general principle in the attribution system, and the principle of presumption of fault and the principle of no-fault liability are applied only in statutory circumstances. If the principle of fault liability is adopted, in the face of the infringement of personal health information, the information subject needs to produce evidence to prove the fault of the infringer. Under the background of the era of medical informatization, the information subject is in a weak position, the status of the information subject and the information collection controller is seriously unbalanced, and there is a big difference in the evidentiary ability of the two sides, so the burden of proof required the information subject is too harsh. In judicial practice, for the sake of protecting personal information, the principle of attribution of responsibility in personal information infringement cases has changed to the principle of presumption of fault, such as the “Pang Lipeng *v*. China Eastern Airlines Co., Ltd. and Beijing Quna Information Technology Co., Ltd. Privacy Dispute Case,” in which the court collected evidence between Pang Lipeng and the defendant company. Considering the extreme asymmetry of ability, it is believed that the law should not require Pang Lipeng to prove that it must be the defendant company that leaked its private information, but that the defendant company should produce evidence to prove that it is not at fault. Since neither company had proven that the disclosure was attributed to other causes, the court found that the two companies were at fault, excluding the possibility of other disclosures of private information. From the perspective of legal provisions, Article 58 of the Tort Liability Law stipulates the principle of presumption of fault in medical damage. Therefore, as sensitive information in personal information, it is feasible to apply the principle of presumption of fault in China.

*(2) Determine the Constituent Elements of Tort Liability*. It is generally believed that the constituent elements of tort liability include the fact of damage, the illegal act, the causal relationship between the illegal act and the fact of damage, and the fault of the perpetrator. For the infringement of personal health information, the illegal acts include two types: acting or not doing. As an act that refers to the perpetrator's initiative to infringe on the right to personal health information of others, it is manifested as an irregular act of collecting, using, and processing, and violating the code of conduct. Inaction refers to the noncooperation of the perpetrator when he or she fails to fulfill his obligation to ensure the safety and security of personal health information and when the information subject exercises the right to correct or block the right, although he or she has not taken the initiative to commit the harmful act. Even if the principle of presumption of fault is stipulated to be adopted for infringement of personal health information, the establishment of tort liability must also meet the fault element, which is only a matter of the allocation of the burden of proof. Due to the prevalence and harmful nature of personal health information infringement, the fact that the composition of personal health information infringement liability requires damage has not yet been determined. The first reading draft of China's Draft Civil Code stipulates that medical institutions and medical personnel who leak patients' personal information and cause damage to patients shall bear tort liability. The second and third reading drafts of the Draft Civil Code delete the provision of “causing harm to patients” and adopt strict liability for the establishment of personal health information infringement, without damaging the facts. Although the Deliberation Draft restricts the infringing subjects and infringements of personal health information, based on the consideration of legislative consistency, the author believes that the constituent elements of personal health information infringement liability do not include the fact of damage, and as long as the perpetrator commits the illegal act and is at fault, the actor should bear the tort liability.

*(3) Determine How to Bear Tort Liability*. According to the provisions of the Tort Liability Law, the methods of bearing the infringement of the personal health information rights of information subjects include nonproperty bearing methods and property bearing methods. Among them, the way to bear nonproperty tort liability mainly includes stopping infringement, removing obstacles, eliminating impacts, etc., such as stopping the collection and processing of personal health information. The property liability method includes property damage compensation and moral damage compensation. The property value and personality value of personal health information provide the basis for the right holder to claim property damages and moral damages. In personal health information infringement cases, the amount of property damages is difficult to calculate, and the author believes that the amount of compensation can be determined according to the order of compensation for “property loses of information subjects—improper benefits obtained by infringers—statutory compensation.” The determination of compensation for moral damages may be determined from the perspective of a “rational person” on the basis of the degree of connection between personal health information and personal dignity.

### 4.5. Introduction of Public Interest Litigation

In the context of medical informatization, cases of infringement of personal health information occur frequently, often on a large scale and in a wide range. Due to the high cost of maintaining rights, many infringed information subjects in practice have not sought judicial remedies. In order to effectively safeguard the lawful rights and interests of information subjects, consideration may be given to introducing the public interest litigation system in the Civil Procedure Law into cases of infringement of personal health information.

Personal health information is of a public interest nature. Researchers in the medical field can promote the development and advancement of medicine by collecting, analyzing, and using personal health information. The improvement of diagnosis and treatment technology and the research and preparation of medical drugs require the use of personal health information. With the help of a large amount of personal health information, the state can carry out public health data monitoring and effectively analyze the health status of the whole people. In practice, a large number of personal health information are used for public welfare, and the public welfare of personal health information is prominent. Therefore, personal health information not only involves the personal interests of information subjects, but also involves the public interest. Public interest litigation mainly targets acts that infringe on the societal public interest, which shows that the introduction of public interest litigation to protect personal health information is reasonable.

In the medical information environment, it is more difficult for individual information subjects to protect their rights. The status, economic strength, and technical ability of health information subjects and information controllers are unequal, and it is difficult for information subjects to effectively safeguard their rights. In addition, information controllers often use personal health information on a large scale, and the number of infringed entities is large and scattered. These characteristics are similar to environmental public interest litigation and consumer public interest litigation. Public interest litigation is litigated on behalf of public interest organizations or corresponding state organs, which can effectively make up for the inequality between information subjects and information controllers, reduce the litigation costs of information subjects, and save judicial resources.

Public interest litigation has the functions of supervision and prevention and protection. Individual information subjects usually become aware of the infringement of their right to personal health information after the damage has occurred, while public interest organizations and personnel are able to detect the illegal conduct of the information controller before the damage occurs. Therefore, the introduction of the public interest litigation system is conducive to solving the problem of personal health information protection from the source.

Personal health information reflects the physiological and mental health conditions of information subjects, and can construct a personal health profile, which contains higher personality value and economic value. With the continuous construction and development of medical informatization, there are problems such as improper collection, improper disclosure, improper use, improper preservation, and other problems of personal health information, the means of infringement continue to escalate, and a large number of cases of infringement of personal health information have emerged. In the dual vortex of big data and risk society, the protection of personal health information is encountering unprecedented problems. Whether it is a unified legislative model based on the right to information self-determination, a decentralized legislative and infringement protection model based on privacy rights, or an industry self-discipline model based on professional ethics, it is impossible to fully respond to the risks faced by personal health information in the big data environment. At present, risk regulation measures that have achieved initial results in areas such as environmental protection and food safety are a good prescription for dealing with the risks of personal health information. Due to the theoretical obstacles encountered by individual responsibility in dealing with risk regulation issues, the use of administrative law methods that are good at collective governance has become an inevitable requirement. The construction of an administrative regulatory system for personal health information risks must closely focus on the two basic issues of science and legitimacy.

## 5. Conclusion

In the dual vortex of big data and risk society, the protection of personal health information is encountering unprecedented problems. Whether it is a unified legislative model based on the right to information self-determination, a decentralized legislative and infringement protection model based on privacy rights, or an industry self-discipline model based on professional ethics, it is impossible to fully respond to the risks faced by personal health information in the big data environment. At present, risk regulation measures that have achieved initial results in areas such as environmental protection and food safety are a good prescription for dealing with the risks of personal health information.

## Figures and Tables

**Figure 1:** Features of big data.

**Figure 2:** Typical Internet health service model.

**Figure 3:** The whole process of residents seeking medical treatment.

**Figure 4:** Privacy of personal information data in the field of health care.

**Figure 5:** Personal health information collection of smart wearable devices.

**Figure 6:** Personal health analysis based on user portrait technology.

**Figure 7:** The privacy protection model of medical big data in the whole life cycle.

**Table 1:** Regulations and systems for the protection of personal health information of medical big data.

Type	Content
Law	Article 111 of the Civil Code of the People's Republic of China
	Article 62 of Chapter 7 of the Law of the People's Republic of China on Authorized Responsibilities
	One of Chapter 253 of the Criminal Law of the People's Republic of China
	Chapter 1, Article 4 of the Mental Health Law of the People's Republic of China
	Article 42, Paragraph 6, of the Law of the People's Republic of China on Administrative Penalties for Public Security
	Article 34 of the Maternal and Child Health Care Law of the People's Republic of China
	Article 23, Paragraph 3 of the Medical Doctor Law of the People's Republic of China (effective as of March 1, 2022) Article 12 of the Law of the People's Republic of China on the Prevention and Control of Infectious Diseases
	Article 22 of the Cybersecurity Law of the People's Republic of China
	Article 38 of the Data Security Law of the People's Republic of China

Administrative regulations	Article 39 of the Regulations on AIDS Prevention and Control

Ministerial regulations	Regulations on the Administration of Medical Records in Medical Institutions (2013 Edition)
	Standard for the Application and Management of Electronic Medical Records (trial)
	National measures for the management of big data standards, safety and services of health care (trial) measures on the management of population health information
	Technical Guide for the Construction of Telemedicine Information System
	“The technology of data management in Linwei test is in southern China)”

National standard	Code for Personal Information Security of Information Security Technology
	Health Informatics Guidelines for Data Protection for the Cross-border Flow of Personal Health Information Information Security Technology Personal Information Security Impact Assessment Guide)
	(“Information Security Technology data fill out Security Assessment Zhainan (Grass Room)”)
	“Information security technology personal information de-identification Zhainan”
	“Information Security Technology, Health and Medical Information Security in South China”

Guiding document	“outline of” healthy China 2030″ Plan
	“guiding opinions on promoting and standardizing the Application and Development of big data in Health Medical Care” on promoting the Development of Internet + ‘s Medical Health

## Data Availability

The labeled data set used to support the findings of this study is available from the corresponding author upon request.
